The article "Effect of Multimedia Health Education on Psychological Burden, Quality of Life Ability, and Self-Efficacy of Congenital Microtia" was published in 2022. Journal: Comput Math Methods Med.

# Effect of Multimedia Health Education on Psychological Burden, Quality of Life Ability, and Self-Efficacy of Congenital Microtia

**DOI:** 10.1155/2022/1482865

**Published:** 2022-08-11

**Authors:** Yanni Zhou, Xiaoxia Li, Meiyi Zhang, Guifen Lv, Bing Duan, Zhujun Tang

**Affiliations:** Department of Plastic and Cosmetic Surgery, Nanfang Hospital, Southern Medical University, Guangzhou, 510515 Guangdong Province, China

## Abstract

**Aims:**

To investigate the effects of multimedia health education on psychological burden, quality of life, and self-efficacy of patients with congenital microtia.

**Materials and Methods:**

Eighty cases of patients with congenital microtia treated and cared for in our hospital from June 2018 to June 2022 were selected according to the numerical table method as retrospective study subjects and divided into 40 cases each in the comparison group and the observation group. The comparison group implemented conventional health education and discharge instruction, and the observation group implemented multimedia health education care to compare the effects of self-efficacy, self-care ability and psychological burden of patients in the two groups.

**Results:**

Before care, the two groups had no statistically significant difference in the quality of life scores (*P* > 0.05). Aftercare, the mental vitality scores, social interaction scores, emotional limitation scores, and mental status of patients in the observation group were significantly higher than those in the comparison group (*P* < 0.05). Before nursing care, there was no statistically significant difference in the nursing ability and anxiety-depression scores between the two groups (*P* > 0.05). After nursing care, the health knowledge level, self-care skills, self-care responsibility, and self-concept of the observation group were higher than the comparison group, while the depression-emotional disorder scores were significantly lower than the comparison group (*P* < 0.05).

**Conclusion:**

Routine health education and discharge instruction combined with multimedia health education care can effectively improve the quality of life of patients with congenital microtia, reduce adverse emotions, and improve patients' sense of self-efficacy.

## 1. Introduction

Congenital craniofacial malformations refer to deformities of the skull, orbit, cheekbones, jaws, and facial soft tissue defects caused by genetic abnormalities or abnormal embryonic development, often accompanied by dysfunction of the five senses [1]. Clinically, congenital craniofacial malformations are generally divided into cranial suture premature autism, craniofacial fissure, facial asymmetry, orbital distance widening, and craniofacial deformity-related syndromes according to clinical manifestations and anatomical sites [2]. Congenital microtia is a morphological malformation of the auricle, often accompanied by atresia of the external auditory canal, hypoplasia of the middle ear, or concurrently with a maxillofacial malformation on the affected side, which is the second most common craniofacial congenital malformation after cleft lip and palate, with an incidence of approximately 3.06 per million newborns in China [3]. The clinical manifestation is the partial or complete loss of the basic structures of the auricle, with only residual auricular cartilage and part of the earlobe, which causes a serious burden for patients and their families [4]. Its causative factors are mostly related to viral infections, medications, and preeclampsia in women in early pregnancy [5]. Microtia is not only a cosmetic and appearance defect but also seriously affects the development of the patient's physical and mental health [6]. Most patients begin noticing their childhood physical defects, leading to dissatisfaction with their body image. Excessive attention, ridicule, and mockery of their surroundings can cause varying degrees of psychological impact and psychological problems [7]. However, with regard to the psychological impact of congenital defects in patients with microtia, the ability of patients with microtia to have a positive state of mind is not only related to whether the surgery can be performed successfully and the degree of satisfaction after surgery, but also to the future healthy development of the body and mind of patients with pediatric malformations [8]. Therefore, studying the psychological problems of patients with microtia helps the smooth operation and is important for promoting the physical and mental health of patients with microtia.

The article "Effect of Multimedia Health Education on Psychological Burden, Quality of Life Ability, and Self-Efficacy of Congenital Microtia" was published in 2022. Journal: Comput Math Methods Med.

Multimedia health education presents the links between knowledge in an organized, hierarchical, and radial manner, including the use of illustrations, cartoon pictures, and words [9]. The complex and disordered thought process is presented with simple and clear pictures to visualize the complex implicit knowledge to some extent [10]. Patients can reintegrate information through multiple perceptions, such as visual-auditory, to strengthen the imaginative connection between the word picture and the brain, thus improving the healthy development of the mind and body [11]. Our study investigated the effects of conventional health education and discharge instruction combined with multimedia health education care on self-efficacy and adverse emotions in patients with congenital microtia, providing some reference basis for clinical care of congenital microtia.

## 2. Methods

### 2.1. Research Object

Our study included information from patients' medical records for the study, complying with the principle of personal information protection, without the need for ethical approval documents nor informed consent from patients and families. Eighty patients with congenital microtia treated and cared for in our hospital from June 2018 to June 2022 were selected as retrospective study subjects according to the numerical table method. Patients with congenital microtia who met the inclusion criteria were numbered according to the order of care and randomized into 40 cases each in the comparison and observation groups using the numerical table method of the third edition of Medical Statistics [12]. The diagnosis of congenital microtia was in accordance with the diagnostic criteria of the “Principles of Diagnosis and Treatment of Congenital External Middle Ear Malformation Syndrome” [13]. Marx classification are as follows: degree I: the size and shape of the auricle are mildly mutilated, slightly smaller than the normal ear, but important surface marker structures of the auricle exist, only slightly structurally altered, with a small auricular cavity and canal opening; degree II: most structures of the outer ear are not recognizable, and the mutilated ear is irregular, peanut-shaped, salami. In degree II, most of the structures of the outer ear are not recognizable, and the residual ear is irregular, peanut-shaped, salami-shaped, etc., and the external auditory canal is often atretic. All patients completed the study, and no patients dropped out of the study halfway through.

### 2.2. Inclusion and Exclusion Criteria

Inclusion criteria are as follows: (1) all selected patients had not received health education, and all selected patients were of normal intelligence and had no other diseases; (2) patients were >5 years old, had their first general anesthesia surgery with postoperative placement of a central negative pressure drain, and all had at least 1 accompanying family member; (3) patients and family members were well compliant, patients were adult patients, and patients and/or accompanying family members were informed about this study; (4) clinical information about patients were complete. Exclusion criteria are as follows: (1) those with other types of diseases, such as endocrine diseases and cardiovascular diseases; (2) those with psychiatric disorders, such as depression and bipolar disorder; (3) those with severe combined trauma, such as severe cranial injury and thoracic and lumbar fractures, history of drug allergy, and history of major surgery; (4) people with other ear deformities; and (5) patients who suffered a postoperative ear impact and injury.

The article "Effect of Multimedia Health Education on Psychological Burden, Quality of Life Ability, and Self-Efficacy of Congenital Microtia" was published in 2022. Journal: Comput Math Methods Med.

### 2.3. Routine Health Education and Discharge Instructions

In the comparison group, routine health education and discharge instructions were applied, and patients and their families were given a discharge education sheet to inform them of the precautions to take. Routine health education and discharge instructions were applied. Specifically, these include the following: (1) patients of the same procedure (younger patients were replaced by their parents) were organized in a quiet ward with a discharge mission sheet and pen for each person, and the time of stitch removal was informed and recorded for them. (2) The missionary nurse is familiar with the contents of the postoperative missionary education for external ear reconstruction and is proficient in handling procedures, methods, and techniques. The nurse assumed the role of the facilitator and first asked the patient or family to read the homemade health education form in our department. The patient had a basic knowledge of discharge education and external ear care by reading it. In order to strengthen the patient's impression, the nurse then asks the main questions to check whether the content of the mission sheet is understood. (3) The patient is asked to ask the nurse questions about the details of various aspects of the health mission sheet that are not understood. The nurse patiently and carefully provides answers to the questions, such as the dose and frequency of oral medication; the method of applying scar removal medication; and wearing ear muffs to protect the ear during children's outdoor activities. When a patient or family member asks a question, the nurse should provide a detailed answer, inform them of the key points and precautions for postoperative care, and give them a positive evaluation of their question. (4) The nurse should ask only one patient to ask a question at a time. When two or more patients ask a question, the nurse asks the unasked patient to record his question to be answered in detail in the next session. (5) The time limit is 20~25 min, sometimes extended by 5 min for better results. At the end of the study, patients (or family members) fill in the health education knowledge assessment form to check the learning results.

### 2.4. Multimedia Health Education Care

In the observation group, multimedia health education nursing was implemented on this basis. The content of preoperative health education was discussed and completed by all nurses according to the actual situation of the department and the disease. Multimedia was made through pictures, texts, sounds, and images, and for the characteristics of the general young age of patients, some cartoon pictures and words were used to make the young children easy to understand and accept, and the duration was about 15 min. (1) The number of patients who have completed the operation and the results of the operation. (2) Preoperative preparation. It includes instruction on fasting and abstaining from drinking to prevent aspiration pneumonia and ventricular rest due to anesthesia or intraoperative vomiting; instruction on improving all relevant examinations to prepare the patient for the surgical procedure; and instruction on personal hygiene preparation for the patient. (3) Respiratory function exercise. Instruct the patient to perform effective coughing and coughing exercises. Since the rib cartilage is to be removed from the chest, teach the patient to press the wound with his hand when coughing to prevent the wound from splitting due to excessive force when coughing. (4) Care of drainage tube. After the operation, negative pressure drainage was left in the ear for 7 d. Patients were instructed to move gently in bed and not to fold and pull the drainage tube, and children should be prevented from grasping and pulling to avoid accidental extubation. (5) Diet and psychology. Instruct the patient to maintain an optimistic and positive attitude, and eat a high protein, high vitamin, and easy to digest diet to ensure postoperative nutrition and calorie supply. (6) Accompanying visitation and management. To ensure orderly medical care, implement the “one patient, one escort” system. (7) After the completion of the education, the multimedia education content can be copied and repeatedly played on the television set in the ward to strengthen the understanding and memory of the children and their families. (8) Self-concept. Patients are prone to questioning, anxiety, and panic due to the lack of basic knowledge of the disease and surgical treatment. The nursing staff should explain to the patients at least once every 4 days for at least 30 min about the disease, surgery, and nursing care and the necessity of implementation to alleviate their negative emotions and promote the improvement of patient cooperation. Before the operation, patients were introduced to knowledge about the operation by means of video or text and were informed of the possible complications and risks associated with the operation and were informed of the relevant precautions so that they could have a clear idea of what to expect and reduce their nervousness and anxiety. Answer patients' questions carefully and try to meet their reasonable psychological needs. The patient should also be instructed to train the pelvic floor and abdominal muscles and be informed of the importance of training to improve compliance. (9) Mutual trust. Patients are easily affected by medical instruments, environment, various invasive operations, and medications during hospitalization, which may result in irritability and disgust and reduce their treatment compliance. Therefore, medical staff and family members should give more emotional support to patients to promote their sense of security, and nursing staff should use easy-to-understand language and be sincere and friendly when communicating with patients to enhance patients' goodwill and improve their treatment compliance. (10) Role function. Patients will impact their emotions due to pain. Nursing staff should give encouragement and comfort to patients, encourage them to tell their true feelings and do a good job in their thinking, and tell their families to care more about the patients to help them face the disease positively.

The article "Effect of Multimedia Health Education on Psychological Burden, Quality of Life Ability, and Self-Efficacy of Congenital Microtia" was published in 2022. Journal: Comput Math Methods Med.

### 2.5. Observation Index

Our study was followed up for 1 month without withdrawal, and the effects of self-efficacy, nursing competence, and dysphoria were observed in both groups before and aftercare. (1) For self-efficacy, the self-efficacy scale (CPSS) was used to assess the self-efficacy of the two groups of hemodialysis patients aftercare, which consisted of three dimensions: somatic function, pain management, and symptom coping, and the higher the score value, the stronger the self-efficacy of the patients. The internal consistency reliability coefficient of the scale was 0.896, the Guttmann score reliability was 0.763~0.896, and the retest reliability was 0.810~0.902. (2) In quality of life score, including mental vitality score, social interaction score, emotional limitation score, and mental status score, each part was scored 0-100, and the higher the score, the better the quality of life of the patients with broken finger reimplantation. (3) Self-care ability assessment scale includes 46 items in 4 dimensions, namely, health knowledge level (14 items), self-care skills (12 items), self-care responsibility (8 items), and self-concept (9 items). Each item is scored 5 points, of which 11 items are reverse scored out of 172 points, the higher the score the better the self-care ability. (4) The anxiety and depression self-assessment scale (SAS) was used to assess the anxiety changes in both groups. (5) Depression self-assessment scale (SAS) contains 20 items with scores from 0 to 100; below 50 is normal; the higher the score, the more serious the patient's depression. The above scales were measured before use with a Cronbach's alpha value greater than 0.914. Patients completed the test independently without any internal or external factors, and the test was completed within 60 minutes.

The article "Effect of Multimedia Health Education on Psychological Burden, Quality of Life Ability, and Self-Efficacy of Congenital Microtia" was published in 2022. Journal: Comput Math Methods Med.

### 2.6. Statistical Analysis

All statistical data in this study were entered into excel software by the first author and the corresponding author, respectively, and the statistical processing software was SPSS25.0 for calculation. Repeated measures analysis of variance between groups was used to measure the measurement expressed as mean ± standard deviation ($\bar{x}\pm \text{SD}$). *χ*2 tested count data are expressed as a percentage (%). The risk factors with significant differences were screened. Included data that did not conform to a normal distribution was described by *M*(QR), using the Mann–Whitney test. The statistical significance was *P* < 0.05.

## 3. Results

### 3.1. Comparison of General Information

The gender, age, and body mass index of the patients in the observation group were similar to those in the comparison group, and the difference was not statistically significant (*P* > 0.05), which was comparable. See Table 1.

### 3.2. Self-Efficacy Comparison

Before nursing, there was no significant difference in the quality of life scores between the two groups (*P* > 0.05). After nursing, the physical function score, pain management score, and symptom coping score of the observation group were significantly higher than those of the control group, and the difference was statistically significant (*P* < 0.05). See Figure 1.

### 3.3. Quality of Life Score Comparison

Before nursing, there was no significant difference in the quality of life scores between the two groups (*P* > 0.05). After nursing, the mental vitality score, social interaction score, affective limit score, and mental status of the observation group were significantly higher than those of the control group, and statistics showed that the difference was statistically significant (*P* < 0.05). See Figure 2.

### 3.4. Anxiety and Depression Score Comparison

Before nursing, there was no significant difference in the scores of anxiety and depression between the two groups (*P* > 0.05). After nursing, the scores of anxiety and depression in the observation group were significantly lower than those in the control group, and statistics showed that the difference was statistically significant (*P* > 0.05). See Figure 3.

## 4. Discussion

As the medical model has changed, the understanding of disease has evolved and deepened [14]. Clinical studies have found that material factors may lead to physical and psychological disorders, while psychological factors can cause physical and mental disorders [15]. In today's material living standards, in the society where mental pressure has a greater and greater impact on human beings, healthy psychological development is crucial to people's lives [16]. Congenital microtia not only affects the patient physically, but also the state of psychological [17]. Psychological problems is a series of problems caused by the inner mental factors of the person, the central nervous control system of the brain, which can indirectly change the personality, world view, and emotions of the person [18]. It can be manifested in life and work as maladjustment, incongruity, and distress, which affects normal life, learning, and work [19]. The factors of mental ill health include biological, psychological, and sociocultural factors [20]. Biological factors are mental health problems caused by genetic, brain, personality, age, and physical damage, and psychological factors are due to changes in the social environment that affect the functioning of the body through psychological and behavioral abnormalities, such as stress and life events and natural disaster factors [21]. Psychologists have shown that biological factors determine the occurrence and existence of psychological phenomena and social factors and the direction of occurrence, development, and change of psychological phenomena [22]. Social factors include environmental, cultural, economic, moral, and educational levels [23].

The article "Effect of Multimedia Health Education on Psychological Burden, Quality of Life Ability, and Self-Efficacy of Congenital Microtia" was published in 2022. Journal: Comput Math Methods Med.

In our study, patients were first informed about the causes of their negative emotions such as anxiety and depression, and then stimuli favorable and unfavorable to recovery were identified. In the intervention phase, specific interventions such as health education, diversified communication activities, and targeted counseling were carried out according to the different characteristics of the patients in order to achieve a good psychological state and improve depressive symptoms [24]. The nursing staff assessed the main psychological and physiological cognitive interventions of the patients, identified the influencing factors associated with them, and developed a targeted care plan for the patients, thus helping them to alleviate their psychological condition and promote their psychological adaptation [25]. The use of multimedia health education in the treatment of many diseases has been reported to have positive implications for improving patients' attitudes and treatment outcomes [26].

In our study, the somatic function score, pain management score, and symptom response score of self-efficacy of patients in the observation group were significantly higher than those in the comparison group aftercare, indicating that conventional health education and discharge instructions combined with multimedia health education care can effectively improve the self-efficacy of patients with congenital microtia. The reasons for this are as follows: self-efficacy is related to the individual's psychological expressions of self-confidence, anxiety, depression, helplessness, and fear when facing various external environments [27]. Self-efficacy is the judgment and speculation of an individual about his or her ability to perform a certain behavior and is a determinant of the human body's ability to perform certain behaviors [28]. A person with a strong sense of self-efficacy is confident in all difficulties, i.e., the stronger the patient's sense of self-efficacy, the better his or her confidence in disease treatment, and the higher his or her compliance with treatment and care implementation [29]. By strengthening communication and exchange with patients, patiently listening to what they have to say, carefully answering their questions, and providing correct guidance, nursing staff promote a cordial nurse-patient relationship and relieve patients' psychological burden [30]. The encouraging language was adopted to enhance their confidence in overcoming the disease, explain their condition to the patients carefully, explain patiently, correct the patients' previous misconceptions of cognition, and guide how to carry out the correct way of coping [31]. Successful clinical cases were used to encourage patients and instruct them to adjust their lifestyle, develop good habits, and perform regular exercise routines, thereby improving their sense of self-efficacy [32]. It can be seen that improving patients' self-efficacy is extremely crucial to accelerate their recovery.

The article "Effect of Multimedia Health Education on Psychological Burden, Quality of Life Ability, and Self-Efficacy of Congenital Microtia" was published in 2022. Journal: Comput Math Methods Med.

The mental vitality score, social interaction score, emotional limitation score, and mental status of patients in the observation group were significantly higher than those in the comparison group after our study care, indicating that conventional health education and discharge instruction combined with multimedia health education care can effectively improve the quality of life of patients with congenital microtia. By carrying out conventional health education and discharge instruction combined with multimedia health education nursing intervention, the patients' poor cognition was changed, and cognitive reconstruction was carried out [33]. Patients were made to consciously discard unstable factors in their daily life, adopt relaxation techniques to effectively cope with stress in all aspects, and then establish a healthy behavior and psychological approach to effectively improve the quality of life of patients [34].

The level of health knowledge, self-care skills, sense of self-care responsibility and self-concept in the observation group were higher than those in the comparison group after our study care, while the depressive mood disorder scores were significantly lower than those in the comparison group, indicating that conventional health education and discharge instruction combined with multimedia health education care can effectively improve the self-care ability of patients with congenital microtia. This may be related to the following advantages of multimedia health education: patients' physiological and psychological adaptation mechanisms are strengthened, their adaptation range is expanded, and their tolerance to stimuli is subsequently increased [35, 36]. Multimedia health education is good control of the primary and secondary stimuli relevant to the patient, keeping the adaptation of the patient's body within its acceptable range and thus avoiding or minimizing the impact of adverse stimuli on the organism [37]. Individual support and encouragement mechanisms implemented during care can help patients to face the stimuli correctly so that individual adaptive responses can be enhanced and maintained, thus promoting the improvement of patients' dysphoria and enhancing self-care and self-efficacy [38].

The article "Effect of Multimedia Health Education on Psychological Burden, Quality of Life Ability, and Self-Efficacy of Congenital Microtia" was published in 2022. Journal: Comput Math Methods Med.

Our study is innovative and has some limitations. First, our study included congenital microtia patients without routine health education and discharge instruction combined with multimedia health education care to assess self-efficacy and poor mood in congenital microtia patients. Second, the selected patients were all from patients treated or cared for in our hospital, so the selection of included and excluded patients was subjective, and the study results may not be representative or biased. Finally, our study only investigated the effect of conventional health education combined with multimedia health education care on self-efficacy and poor emotion in patients with congenital microtia and failed to study patients with congenital microtia in depth and follow up their recovery after congenital microtia care for a long time.

## 5. Conclusion

Conventional health education and discharge instruction combined with multimedia health education care can effectively improve the quality of life of patients with congenital microtia, reduce adverse emotions, and improve patients' self-efficacy, which has certain reference value for the care of patients with congenital microtia.

## Figures and Tables

**Figure 1:** Self-efficacy comparison. (a). Physical function score; (b) pain management score; (c) symptom coping score (values expressed as mean ± standard deviation). ^∗^*P* < 0.05 vs. control group.

**Figure 2:** Quality of life score. (a) Mental vitality score; (b) social interaction score; (c) affective limit score; (d) mental status scores (values expressed as mean ± standard deviation). ^∗^*P* < 0.05 vs. control group.

The article "Effect of Multimedia Health Education on Psychological Burden, Quality of Life Ability, and Self-Efficacy of Congenital Microtia" was published in 2022. Journal: Comput Math Methods Med.

**Figure 3:** Anxiety and depression score. (a) Anxiety scores; (b) depression scores (values expressed as mean ± standard deviation). ^∗^*P* < 0.05 vs. control group.

**Table 1:** Comparison of general data between the two groups [*n*, ($\bar{\chi }\pm s$)].

Group	Age (years)	Sex (male/female)	Body weight (kg)	Marx		
				I	II	III
Observation group (40)	9.48 ± 1.37	13/27	23.33 ± 2.51	10	19	11
Comparison group (40)	9.93 ± 1.19	14/26	23.32 ± 2.59	11	17	13
*χ* ^2^/*t*	-1.568	0.056	0.018	0.313		
*P*	0.161	0.813	0.986	0.855		

## Data Availability

The datasets used and analyzed during the current study are available from the corresponding author upon reasonable request.
